RETRACTED

# Construction of Financial Management Early Warning Model Based on Improved Ant Colony Neural Network

**DOI:** 10.1155/2021/6748920

**Published:** 2021-11-23

**Authors:** Meiluan Wang

**Affiliations:** Department of Accounting, Zhejiang Gongshang University, Hangzhou, Zhejiang 310018, China

## Abstract

With the advent of the era of economic globalization, the world capital market is also facing financial risks. It is necessary to have a corresponding financial management early warning model to reduce economic losses. This paper uses the combination of ant colony algorithm and neural network algorithm to build a neural network improved by ant colony algorithm model. By setting relevant assumptions, the financial statements and annual report texts are predicted and analyzed and compared with the original static data forecasting model. Compared with traditional methods, the time series sequencing analysis used in this paper makes the result prediction more accurate. This allows one year's data to be used to predict the data for the next two years. This research can provide a corresponding reference for the optimization of financial management early warning system.

## 1. Introduction

The annual report is one of the inspections that enterprises need to handle every year. In short, the annual report is that the operating enterprises copy the annual report to the industrial and commercial authorities through the market subject credit information publicity system and publicize it to the society. Many bosses may say that it is troublesome to do this once a year. Is it necessary to do it every year? In fact, in addition to the mandatory provisions, the annual report is also good for enterprises. Through the enterprise credit information publicity system, the annual report is directly submitted to the administrative department for industry and commerce, which is conducive to confirming the business qualification and business ability of the enterprise. The enterprise information publicity system helps to strengthen the supervision and management of enterprises, plays a certain role in deterrence and inventory, and protects the legitimate rights and interests of enterprises. The relevant departments also have strict requirements on the accuracy and integrity of the publicity of enterprise annual inspection information. Any enterprise that makes a false report or fails to report may be listed in the list of abnormal operations by the Administration for Industry and Commerce.

The annual report of an enterprise has always been one of the important references for stakeholders to invest, and it is also an important source for the public, investors, and trading counterparts to understand the enterprise information. When the public has no more channels to understand a company, they will look for the annual report of the company to read and make investment decisions according to their own experience. In 1932, after the first economic crisis, Fitzpatrick paired samples of bankrupt enterprises and nonbankrupt enterprises, which opened the history of quantitative analysis of financial early warning. These 19 pairs of samples were divided into two groups based on the single variable financial ratio index. Finally, it was found that the two indexes with the strongest ability to predict the financial crisis were return on equity, shareholders' equity, and liabilities [1]. In 1986, with the rapid development of computer technology, some people began to try to study a large number of samples. Beaver made an empirical study with the same idea as Fitzpatrick and compared a large number of companies with normal financial situation and financial crisis. Finally, another powerful indicator for financial crisis prediction was found: the ratio of cash flow to total liabilities [2]. For a long time, the main research method of this problem is univariate analysis. Until 1968, Altman put forward a landmark new practical model, namely, five-variable Z-score model, which opened the era of using multivariate statistical methods to predict financial crisis [3]. The Z-score model selects 22 financial index data and makes a comparative analysis on the prediction variable “whether the company has bankruptcy risk,” which has achieved good results and has been widely used in Europe and the United States.

RETRACTED

Based on the previous literature review, this paper determines the purpose and method of this study, that is, using the data of financial statement indicators and the body of the annual report to predict the problem of “whether the listed company is specially treated” and using the neural network improved by ant colony algorithm to predict and analyze it, respectively. An improved ant colony algorithm neural network model is established by innovatively using the combination of ant colony algorithm and neural network algorithm. By setting relevant assumptions, the text of financial statements and annual reports is predicted and analyzed and compared with the original static data prediction model, using time series. This makes the financial company's forecast more accurate. The data of one year can be used to predict the data of the next two years.

This paper is divided into five parts. The first part is the research background. The second part is the literature review, analyzing the research results of the problem. The third part is the introduction of neural network improved by ant colony algorithm. The fourth part is the specific experimental analysis. This part expounds the application of the improved neural network ant colony algorithm in financial management early warning. The fifth part is the conclusion of the article.

RETRACTED

## 2. Related Work

Around 1980, the trend of using machine learning method for classification prediction came, and some people began to apply the early machine learning algorithms such as logistic regression, support vector machine, and artificial neural network to the research of financial crisis early warning, and the sample size of the model was further expanded. Giatrakos et al. used the sample data of more than 2000 bankrupt enterprises and nonbankrupt enterprises to describe the probability distribution of bankruptcy. The logistic regression model was applied to the risk prediction for the first time, and the output value was conditional probability. The higher the probability, the greater the risk of bankruptcy. Finally, the study found four new indicators with strong forecasting ability, namely, total assets, asset liability ratio, financing ability, and profitability [4]. Logistic regression model is simple, fast, and of low data requirements, soon replaced the Z-score model into the industry, has become the mainstream method of risk prediction, and has been used up to now. Subsequently, scholars began to expand horizontally and vertically around multiple logistic regression. For example, Sun et al. substituted the variables of cash flow statement into logistic regression model for analysis and found that capital expenditure and shareholder interest distribution have strong early warning ability [5]. Maheshwari et al. introduced the artificial neural network for the first time to learn the model of 65 pairs of bankrupt and nonbankrupt companies. The input variables of the neural network adopted the characteristics of the commonly used Z-score five-variable model that had been developed and matured at that time. Even if the problem of neural network algorithm solution had not been solved at that time, the model finally achieved 80% accuracy [6]. Yang and Wang used support vector machine to conduct bankruptcy early warning research on bank financial data samples and empirically tested the effectiveness of its application in this field by comparing and analyzing various previous machine learning models [7].

Financial crisis early warning research lags behind other countries. Various research results have been published since around 1990, because financial market has developed rapidly since then. Fortunately, there is a large amount of research literature from other countries as the basis. Research does not need to start from scratch. Most of the research work is to improve the previous model from two aspects: variables and methods. Marinakis believed that the previous models did not fully consider the generalization ability in the actual prediction process, redefined the misjudgment rate, and conducted an empirical study on 20 groups of listed company samples whether they were specially treated. The results show that the effect of support vector machine is significantly due to linear regression and logical regression [8]. Mikalef et al. proposed the PCA-SVM model to predict the financial distress of listed companies and used the principal component analysis method to screen and combine the data characteristics, which improved the prediction effect of SVM [9]. Researchers no longer focused on the improvement of methods and variables but began to apply the model to more subdivided industries. Roth et al. studied the financial crisis of listed commercial banks and found three variables with significant impact: asset quality, financial leverage, and financial change trend [10]. Koppe et al. introduced the *Z*-value multiple linear discriminant method into the field of financial early warning [11]. Stergiou et al. found that the accuracy of multivariate decision model was higher than that of logistic model when the data met the normal distribution, and the accuracy of logistic model was higher than that of multivariate decision model when the data did not meet the normal distribution [12].

RETRACTED

Bibault et al. applied the artificial neural network model to the field of financial distress and proved that the accuracy of the artificial neural network model is higher than that of the multivariate discriminant method [13]. Artificial neural network model can solve the nonnormal distribution and nonlinear problems of experimental data in financial early warning model and reduce the error through a large number of repeated learning data. The artificial neural network model has been widely developed and used [14]. Avci et al. proposed the construction of neural network early warning system [15]. Lv et al. established the financial early warning model of listed companies by using BP neural network model and conducted empirical analysis with 30 training samples and 8 test samples [16]. The accuracy of the final model was 95%. Johnson and Khoshgoftaar used *Z*-value analysis method, logistic regression model, and BP neural network model to model and analyze 100 training samples and 50 test samples, which proved that the accuracy of artificial neural network was higher than the other two models [17]. So far, all the BP neural network models mentioned above are general neural network models, and the optimization algorithm is not used to optimize the model, so there are some limitations. Wang et al. took 60 enterprises in the logistics industry as the training sample data to model and analyze the RBF neural network model and used particle swarm optimization algorithm to optimize the parameters of the neural network. The final accuracy of the model was 83% [18].

RETRACTED

In terms of earnings management, Hou et al. took 6913 listed companies as research samples and proved that 15% of the companies and 53% of the companies in the loss sample would conduct earnings management [19]. Chen took 267 companies as samples and proved that the accuracy of financial early warning model can be improved from 68.9% to 71.9% by considering earnings management factors [20]. Wu et al. conducted a study on 8404 samples of listed companies. The results show that the higher the degree of accrual earnings management, the greater the possibility of financial crisis [21]. Li et al. used the decision tree of tree model as the basic classifier of crisis prediction problem and used the “bagging integration method” to conduct empirical research on manufacturing enterprises, which improved the accuracy of the results and the recognition rate of the model for financial crisis enterprises [22].

Song and Li used descriptive statistics to analyze the situation of information disclosure in the annual reports of companies trading in Shanghai Stock Exchange and found many problems. They believed that, at that time, the company did not implement the mandatory provisions on controlling information disclosure, the information disclosure power was insufficient, and the auditing standards of accountants and audit bureaus were not unified, and they put forward their own suggestions [23]. Bakker et al. conducted in-depth research on the low quality of the information submitted in the annual report and concluded that the important reason for the problem was that there were no clear regulation and rules and regulations to restrict enterprises at that time [24]. Serrano focused on the information disclosure affecting the annual report [25].

In fact, most of the research results are based on neural network model, and the neural network model has a good effect in early warning. This paper also uses neural network improved by ant colony algorithm to study financial management early warning.

## 3. Construction of Financial Management Early Warning Model Based on Neural Network Improved by Ant Colony Algorithm

Ant colony algorithm is an evolutionary algorithm inspired by the foraging behavior of ant colony in nature. In the process of ant foraging, in order to find the shortest path from food to nest, ants will transmit information through pheromone [26]. Each ant leaves pheromone in the process of movement and makes path selection according to the pheromone concentration on the path. The probability of ant choosing a path is proportional to the pheromone concentration on the path. Ant colony algorithm is a simulated evolutionary algorithm. Preliminary research shows that the algorithm has many excellent properties. In this paper, the parameters of PID controller are optimized and compared with the results of ant colony algorithm and numerical simulation. Based on ant colony algorithm, the construction of financial management early warning model of neural network is improved [27].

RETRACTED

Let *m* denote the number of ants, *v*_*i*_,  (*i*=1,…, *n*) denote city points, *d*_*ij*_ denote the distance between city *v*_*i*_ and city *v*_*j*_, and *E*_*ij*_ denote the path between city *v*_*i*_ and city *v*_*j*_; then the ant system mainly includes the following steps:

The first step is to initialize the pheromone concentration. The pheromone on each edge is initialized to a small constant, denoted as *τ*_*ij*_(0)=*τ*_0_.
The second step is to initialize the ant position. Place *m* ants randomly in *n* cities, and the taboo table of each ant is the city where the ant is located.
The third step is to select the transfer path based on the transfer probability. During the movement of the ant *k*, the next city to be transferred is determined according to the amount of information on each path and the path information. *p*^*k*^(*i*, *j*) represents the probability that *t* and *k* will transfer from city *v*_*i*_ to city *v*_*j*_ at time, as shown in formula (1):
  (1) $$\begin{array}{c} p_{ij}^{k}\left(t\right)=\left\{\begin{array}{cc} \frac{\tau_{ij}^{\alpha }\left(t\right)\eta_{ij}^{\beta }\left(t\right)}{\sum_{w\in J_{i}^{k}}\tau_{iw}^{\alpha }\left(t\right)\eta_{iw}^{\beta }\left(t\right)}, & j\in J_{i}^{k},\\ 0, & j\notin J_{i}^{k}, \end{array}\right. \end{array}$$
Among them, *τ*_*ij*_(*t*) represents the strong pheromone of the path *E*_*ij*_ from *v*_*i*_ to *v*_*j*_ at time *t*, and *η*_*ij*_(*t*) represents the path *E*_*ij*_ information at time *t* (TSP is defined as 1/*d*_*ij*_); the parameters *α* and *β*, respectively, represent the degree of influence of the pheromone and path information on the transition probability. *J*_*i*_^*k*^ is the feasible solution domain of ant *k* at city *v*_*i*_, *J*_*i*_^*k*^={1,…, *n*} − tabu_*i*_^*k*^. The artificial ant colony algorithm has a memory function. The set tabu_*i*_^*k*^,  (*k*=1,…, *m*) represents the city that the ant tabu_*i*_^*k*^ has traveled when it reaches the city, and pp will dynamically adjust with the ant's search process.
The fourth step is to update the pheromone. After all the ants have found a legal path, they update the pheromone, and the pheromone on each path is adjusted according to formula (2):
  (2) $$\begin{array}{c} \tau_{ij}\left(t+n\right)=\left(1-\rho \right)\tau_{ij}\left(t\right)+\sum_{m}\Delta \tau_{ij}^{k}, \end{array}$$
Among them, *ρ* ∈ (0,1) represents the pheromone volatilization coefficient, and ∑_*m*_Δ*τ*_*ij*_^*k*^ represents the increase of pheromone remaining on the path by all ants that have gone through the path *E*_*ij*_ in this cycle, and Δ*τ*_*ij*_^*k*^ can be calculated according to formula (3):
  (3) $$\begin{array}{c} \Delta \tau_{ij}^{k}=\left\{\begin{array}{cc} \frac{Q}{L_{k}}, & \text{If the ant is passed }\left(i,j\right),\\ 0, & \text{otherwise}, \end{array}\right. \end{array}$$
Among them, *Q* is a constant (representing the total amount of information released by the ants in a cycle), and *L*_*k*_ represents the length of the path taken by the *k* ant in this cycle. The above algorithm is called the ant-cycle algorithm.
In the fifth step, repeat the second to fourth steps, and record the optimal path of *m* ants in each cycle until the algorithm converges or reaches the maximum number of iterations.
If the length corresponding to the current optimal path *π*^*bs*^ is *L*^*∗*^, each cycle pheromone update is performed according to formula (4):
  (4) $$\begin{array}{c} \tau_{ij}\left(t+1\right)=\left(1-\rho \right)\cdot \tau_{ij}\left(t\right)+\sum_{k=1}^{m}\Delta \tau_{ij}^{k}+\Delta \tau_{ij}^{bs},\\ \Delta \tau_{ij}^{bs}=\left\{\begin{array}{cc} \frac{e}{L^{*}}, & \left(i,j\right)\in \pi^{bs},\\ 0, & \text{otherwise}, \end{array}\right. \end{array}$$
where *e* is the number of elite ants in this iteration or a fixed constant, and *L*^*∗*^ is the corresponding length of the current optimal path *π*^*bs*^. The smaller the *L*^*∗*^ is, the more the pheromones will be added to the current optimal path *π*^*bs*^.

Ant colony system improves the ant system mainly in three aspects.

First, when calculating the transition probability of ants, the ant colony system adopts the pseudo-random proportion rule. In the ant colony system, the ant *k* in the *i* city chooses the next city *l* according to formula (5):
  (5) $$\begin{array}{c} l\left\{\begin{array}{cc} \arg\max_{j\in J_{k}}{\left[\tau \left(i,j\right)\right]}^{\alpha }{\left[\varphi \left(i,j\right)\right]}^{\beta }, & \mathrm{if}\;u\leq u_{0},\\ j, & \text{otherwise}, \end{array}\right. \end{array}$$
In the above formula, if *u* > *u*_0_, the ant will select the next city according to the probability transfer formula *p*^*k*^(*i*, *j*), as shown in formula (6):
  (6) i,jk=τi,jαφi,jβ∑w∈JKτi,wαφi,wβ,j∈JK,0,j∉JK.
*u*_0_ is the random number of [0,1] interval. When *u* > *u*_0_, it represents exploratory search in ant system; when *u* ≤ *u*_0_, the expression represents deterministic search, that is, to find the path with the highest probability from the obtained results as a choice.
Secondly, in order to make ants find the optimal solution faster, the pheromone concentration on the current optimal solution path is only updated when the pheromone is globally updated in the ant colony system. The global update rule is formula (7):
  (7) $$\begin{array}{c} \tau_{ij}\left(t+1\right)=\left(1-\rho \right)\cdot \tau_{ij}\left(t\right)+\rho \Delta \tau_{ij},\\ \Delta \tau_{ij}=\left\{\begin{array}{cc} \frac{1}{L^{*}}, & \left(i,j\right)\in \pi^{bs},\\ 0, & \text{otherwise}, \end{array}\right. \end{array}$$
where *ρ* is the pheromone volatilization parameter, *π*^*bs*^ is the current optimal path, and *L*^*∗*^ is the corresponding length of the current optimal path *π*^*bs*^.
Thirdly, the ant colony system adopts the local update rule, which constructs the path and updates the pheromone concentration at the same time. The local update rule is formula (8):
  (8) $$\begin{array}{c} \tau_{ij}\left(t+1\right)=\left(1-\rho \right)\cdot \tau_{ij}\left(t\right)+\rho \Delta \tau_{0}, \end{array}$$
where *ρ* is the pheromone volatilization parameter and Δ*τ*_0_ is the given parameter. When an ant passes through an edge (*i*, *j*) path, the pheromone concentration of the edge is volatilized immediately, which can increase the probability of ant choosing other paths, increase the global search ability of the algorithm, increase the possibility of choosing the path not passing through, and avoid premature convergence to a certain extent. The ant colony algorithm process is shown in Figure 1:

The financial situation of listed companies generally has two aspects: one is the poor operation of the company; the other is the falsification of the company's financial statements. Through the summary of previous empirical research conclusions and theoretical models, we can divide the indicators to predict the financial crisis into six dimensions: solvency, profitability, operating ability, development ability, cash flow analysis, and risk level.

RETRACTED

## 4. Results and Discussion

In linear regression analysis, when there are certain conditions in the experimental data, only the significance test of the regression equation and regression coefficient can not ensure that the selected independent variables are appropriate. At this time, no matter from the perspective of estimating regression coefficient or prediction, the results are not ideal. Therefore, the linear correlation between variables needs to be solved before the test. The neural network improved by the ant colony algorithm first needs to solve the problem of linear correlation between variables. Firstly, the data is standardized, and then the linear correlation coefficient between the independent variables is calculated. The results are shown in Figure 2.

In this figure, blue indicates that the two variables are positively correlated, red indicates that the variables are negatively correlated, and the darker the color is, the greater the correlation is. It can be seen from the figure that most of the independent variables are not correlated with each other, and only a few of them have high correlation, so the indicators are further screened. *X*1, *X*2, and *X*3 are current ratio, quick ratio, and cash ratio, respectively, which have strong positive correlation. *X*5 is “the ratio of net cash flow from operating activities to current liabilities,” which has strong negative correlation with these three variables; only *X*1 is retained. Similarly, after analysis, the 11 variables *X*2, *X*3, *X*5, *x*9, *X*11, *x*14, *x*17, *X*22, *x*24, *x*30, and *x*37 were eliminated, and only 28 independent variables were retained. Then Bartlett sphere test was performed on the sample data, and the results are shown in Table 1:

It shows that the data does not need to be reduced by principal component analysis, so we can use the method of cross validation, according to the principle of ANOVA, select features according to the percentage of fixed intervals, use the decision tree model to predict all features, make performance evaluation, and score each feature. The change of AUC with the proportion of feature selection is shown in Figure 3:

It can be seen from Figure 3 that the percentage of optimal feature number is 61%, so the optimal feature number is 33 ∗ 61% = 20.13. There are 20 optimal feature variables selected and retained finally. The results show that using the decision tree model to predict all features, evaluate the performance, and score each feature has a good effect. The feature dimension score of the 20 best variables is the highest. According to the scoring results of feature dimension, the 20 variables with the highest score are quick ratio, ratio of total profit to EBIT, return on assets, business cycle B, cash flow of the company long-term return on capital, asset liability ratio, accounts receivable turnover B, Herfindahl_5 index, return on investment, ratio of net cash flow from operating activities to total liabilities, separation of two rights, return on invested capital, operating index, operating gross margin, financial leverage, capital accumulation rate B, net profit, net cash content, growth rate of owner's equity B, and ratio of asset impairment loss to operating income.

RETRACTED

The three models are all learned by Python's sklearn library. When the default parameters of logistic regression are used, the default training iterations are updated 25 times. However, the model cannot converge at this time, so the number of iterations is increased to 100 times. The confusion matrix of the model prediction results obtained on the test set is shown in the following figure.

As can be seen from Figure 4, the number of listed companies that will be specially treated in the test set is 83, and 53 companies have been successfully predicted. The accuracy rate of the model is only 29.77%. That is to say, less than 30% of the listed companies that will be specially treated will really have financial crisis, which may make investors miss many good companies that are developing steadily. The recall rate of the model is 63.85%. This means that 63.85% of the companies with financial crisis risk in the market can be predicted by the model, and the recall rate cannot reach the level of reassuring investors. The accuracy of the model is 89.16%, AUC value is 0.63, *F*1 value is only 0.41, and logistic regression is not good in predicting whether listed companies will be specially treated.

In the learning process of neural network improved by ant colony algorithm neural network improved by ant colony algorithm, AUC value and *F*1 value are used as the measurement standard to observe the change trend of these two evaluation indexes with the number and depth of decision trees in neural network improved by ant colony algorithm. The abscissa and ordinate of Figure 5 represent the number and depth of decision trees, respectively, as shown in Figure 5:

As can be seen from Figure 6, the number of decision trees that make AUC value and *F*1 value reach the maximum at the same time is 5, and the tree depth is 4. The prediction effect of the improved substructure neural network on the test set is as follows.

The results of neural network improved by ant colony algorithm and logistic regression are almost the same, the accuracy is 89.09%, AUC value is 0.64, and *F*1 value is 0.41. When the effect of the two methods is similar and the effect is not good enough, it should be considered that the model selection is wrong or the data has problems; logistic regression and Stochastic Forest belong to linear classifier. This may indicate that the financial data of listed companies are highly uncertain. Although the form is simple, the relationship between them and the financial risk of listed companies is complex and cannot be done with simple linear classifiers. Therefore, we will try to use nonlinear SVM training model next. The training results on the same test set are shown in Figure 7:

The accuracy rate of SVM model is only 34.9%, recall rate is 62%, AUC value is 0.66, and *F*1 value is 0.45, which is better than logistic regression and neural network improved by ant colony algorithm, but it is still not ideal, the early warning effect on investors is very small, and the recognition of companies with financial risks is not high enough. It shows that the relationship between financial data and listed companies is indeed nonlinear, and the data processing method in this paper is not suitable for crisis prediction. In order to achieve better prediction effect, financial data still needs time series data, because the information reflected by the change trend of financial data is more effective than the static information in a certain time section. The amount of information is larger, and the static data may lead to such examples as “the thin camel is bigger than the horse,” which may lead to errors in judging the company's operating conditions only from the numerical value. After that, the forecasting effect of the neural network improved by ant colony algorithm under the time series on the financial crisis will be shown.

RETRACTED

In the previous research on financial crisis prediction based on the annual report of listed companies, sentiment analysis is a very common technology. The tf-idf statistics of positive and negative sentiment words in the annual report is also one of the commonly used indicators to predict financial crisis, and the research results show that this variable is effective. Therefore, this section will show the distribution of emotional words in the samples of positive and negative categories [28, 29].

This paper selects one annual report of listed companies from the positive and negative sample boxes and makes statistical analysis of word frequency according to the dictionary constructed above. Now we import the processed annual report text into *R* and further transform it into structured data suitable for sentiment analysis. We use “tidytext” package text to segment words and then match and count the emotional words in the dictionary. Even if the company's performance is not good enough, such as explaining a certain investment event, a positive sentence such as “the company will actively broaden the financing channels” will be added as a supplement. As a result, if we only look at the number of positive and negative words, it may appear that even if the sample is regarded as having financial crisis, the proportion of positive emotional words is still relatively high. This is also the inadequacy of previous studies. If we only consider the emotional words frequency and other variables extracted from the text, we may lose a lot of key information. This paper adopts the long-term and short-term memory network construction model to explore whether the word order, context, and so on in the annual report text can provide more judgment information.

RETRACTED

Figure 8 is a supplementary illustration, which specifically analyzes the positive and negative emotional words in the annual report of Jinguyuan company and their respective proportions. It can be found from the figure that the word “solve” appears more frequently in the positive vocabulary, which is more like the need to “solve” because of the previous problems. It mainly indicates the signal to reverse the disadvantage and may also indicate the risk of facing problems that cannot be properly solved. The most common negative words are “risk” and “competition.” Generally, the company's current risks will be explained in the annual report. However, companies with relatively stable development or with large market capacity may not be threatened by competition. It can be seen that Jinguyuan company is small in scale and high in risk and the focus of the company's operation is to maintain stability and strive for development. Investors should attach great importance to it.

“*Y* = 1” means that the listed company has been specially treated in this year, and “*y* = 0” means that the financial situation of the listed company in this year is normal and has not been specially treated. The data has been divided into training set, verification set. and test set in advance.

The ant colony neural network selected in this paper is a network structure of 128 neurons. The tool used is the keras Library in Python 3. The iterative epoch = 10 is set at the beginning. The model parameters are updated by small batch gradient descent method, and the number of samples in each batch is set to batch_ size = 16, then the number of trainings needed to complete an epoch is 128, the learning rate is set to lr = 0.001, and the activation function of the output layer is sigmoid.

It can be seen from Figure 9 that, with the increase of the number of iterations, the loss function value of the training set gradually decreases. And the accuracy rate gradually increases, while the loss function value and accuracy rate of the verification set both fluctuate greatly, reaching the minimum value and the maximum value, respectively, in the second iteration and the third iteration, indicating that overfitting occurs when the number of iterations increases. Therefore, epoch = 2 is chosen as the final parameter of the model. It can be found that the comprehensive effect of only two iterations of the model is the best, and the data in the figure shows that, in the first iteration, the loss function value of the data set has been very small, and the accuracy rate has been very high. After analyzing the input vector, the sample size is small, so the number of samples and learning rate of each batch are small, and the training process is more detailed. And the similarity between the input text vectors is high; the cosine similarity of the highest two text vectors is as high as 0.96, which is two samples belonging to the same negative class sample set, indicating that the diversity of input data is low. In this case, it is possible to achieve the best convergence point only by iterating twice. Take epoch = 2 and draw the ROC curve on the verification set, as shown in the figure.

RETRACTED

It can be seen from Figure 10 that when the threshold value is 0.5, the ROC curve on the validation set is drawn as shown in the figure, and the AUC value is as high as 0.98, which indicates that the model has achieved very good prediction results for both positive and negative samples. The sample size of the test set is 723, and the number of companies that have been specially treated (*y* = 1) is 114, 101 of which have been successfully predicted. However, the number of companies not specially treated (*y* = 0) is 609, of which 605 are predicted to be successful.

When the threshold value is 0.5, the accuracy of the model is 97.64%, which is slightly higher than the accuracy of the first model (doc2vec text processing and ant colony neural network model for classification and prediction). The accuracy rate is 96.19%, which is higher than that of the first model, indicating that the early warning effect of the model is better. Among the companies predicted to be specially treated, 96.19% of the companies may really be specially treated, which needs special attention from investors. The recall rate is 88.59%, which is slightly higher than that of the first model. It shows that our model can identify 88.59% of the companies with real financial crisis, and the risk identification ability of the model is also strong. The F1 value and AUC value were 0.92 and 0.93, respectively, which were better than the first model.

## 5. Conclusion

Based on the previous literature review, this paper determines the purpose and method of this study, that is, using the data of financial statement indicators and the body of the annual report to predict the problem of “whether the listed company is specially treated” and using the neural network improved by ant colony algorithm to predict and analyze it, respectively. From the perspective of data, the improved neural network model based on ant colony algorithm based on text data is much better than the model based on financial data, which may be due to the assumption of the relationship between predictive variables and explanatory variables. That is, “securities code + year” is the unique identification of the sample, and the impact of the formed sample on the prediction variables is independent. There is no doubt that considering the change of time series has a greater impact on financial data than not considering the change of time series, but it also shows when the collected samples are limited. The annual report of a certain year can be used to predict whether a listed company will have a special crisis within two years. However, this paper lacks data simulation verification, which needs further explanation in future research.

RETRACTED

## Figures and Tables

**Figure 1:** Schematic diagram of ant colony system.

**Figure 2:** The ant colony algorithm improved neural network algorithm index screening diagram.

**Figure 3:** Broken line graph of AUC ratio change based on neural network improved by ant colony algorithm.

**Figure 4:** Confusion matrix based on financial data in the neural network improved by ant colony algorithm.

**Figure 5:** Changes of AUC and *F*1 values with the number of decision trees (a) and tree depth (b).

**Figure 6:** Confusion matrix of neural network improved by ant colony algorithm model based on financial data.

**Figure 7:** Confusion matrix of support vector machine model based on financial data.

**Figure 8:** Statistical analysis of word frequency in neural network improved by ant colony algorithm.

**Figure 9:** The relationship between the number of iterations of the neural network improved by ant colony algorithm training set and validation set, error value, and accuracy. (a) Training and validation loss. (b) Training and validation accuracy.

**Figure 10:** The roc curve chart in the improved neural network algorithm of ant colony algorithm.

**Table 1:** Bartlett sphere test results of financial index data.

Bartlett sphericity test		
Chi square	*P* value	Conclusion
242.85	1	Unsuited

## Data Availability

The data used to support the findings of this study are available from the corresponding author upon request.
